# Aesthetic and Implication Analysis of the Traditional Poetic Environment Based on Natural Language Emotion Analysis

**DOI:** 10.1155/2022/3300449

**Published:** 2022-09-28

**Authors:** Hui Wang

**Affiliations:** Harbin Normal University, Harbin Far East Institute of Technology, Harbin 150025, China

## Abstract

The uniqueness of aesthetic implication in Zhou Dynasty poetics lies in that it is the basic forming stage of the concept of formal beauty of the whole Chinese nation, and the aesthetic implication of the Zhou Dynasty poetics art has fundamental significance for the whole ancient Chinese aesthetic implication theory. In the discipline of natural language processing, text emotion analysis is a crucial topic. Artificial neural network research is where the idea of “deep learning” (DL) first emerged. In view of the problems that semantic information is easy to be lost and emotional information may be ignored in the traditional Chinese short text emotion analysis model, this paper introduces the AM (attention mechanism) and proposes a CNN-LSTM (convolutional neural network-long short-term memory) poetic aesthetic implication analysis method based on self-attention. For the IL (input layer), word vectors trained by Word2Vec are used and then input into the CNN-LSTM joint model. Then, the output of the joint model is weighted and summed by self-attention and finally input into the Softmax classifier, so as to realize the emotion classification of the text. By creating and putting into practise pertinent comparative experiments, the usefulness of the proposed model is confirmed. The outcomes demonstrate that this model outperforms the other three comparison models for the quantification of evaluation indices in terms of overall performance. The accuracy and F1 of this paper are 93.362% and 90.886%, respectively, which are higher than other models.

## 1. Introduction

The Zhou Dynasty not only liked to use the expression of poetry and prose in daily life but also incorporated the brilliance of poetic thinking in the national governance and the aesthetic value judgment expressed by it. The rites and music system established in the Western Zhou Dynasty were deteriorating day by day, and “the book of poetry” was inevitably affected. There are many words representing cyan in “The Book of Poetry,” but ancient cyan is different from what we call cyan today. What we call cyan today refers to black or dark-blue, while ancient cyan refers to the nascent color of vegetation, which is equivalent to what we call green now. The “music” in the Spring and Autumn period developed from the musical instruments and temperament in the primitive tribal period to the sacrificial music in the Shang Dynasty. Music, as an essential part of sacrificial rites, began to appear on the historical stage, and at the same time, the music among nobles also became popular. In the aesthetic activities and social activities of human beings, the formal factors of things themselves and the displayed combination relations are constantly spreading to people's spiritual and emotional world, thus becoming a necessary existence to satisfy people's lives and emotions.

To explore the ancient people's aesthetics, it is necessary to define a dimension of exploration. Many scholars will explore it from the perspectives of philosophy, art, psychology, ethics, and physiology. The author thinks that the most important thing in aesthetics is humanistic care. The Zhou Dynasty existed for about years, from the middle of the century BC to the year BC, and it was the longest-lasting dynasty in ancient Chinese history. The most notable feature of the Zhou Poetic Culture is the ritual and music system that permeates into social politics and daily life [1]. And “music” was used to carry out the enlightenment idea of the ruling class, which was a great pioneering work of Zhou people. It makes the boring, cold, hierarchical moral, and ethical education become gentle, comfortable, and happy. “The Book of Poetry” is the earliest extant poetry anthology in China, which contains 305 poems from the Western Zhou Dynasty to the middle of the Spring and Autumn period. Each of its works contains countless cultural contents that can be discovered. It provides rich and detailed original materials for us to grasp people's aesthetic notions during that era [2]. It is a pictorial account of ancient Chinese cultural history and a national aesthetic accumulation from ancient society to Zhou culture. This poetic way of thinking about leading the nation through the arts had a significant impact on following generations, developing the idea of poetry and music education and creating China's own ceremonial and musical cultural tradition.

Literature in pre-Qin Dynasty, especially the study of Zhou Dynasty poetics, is often faced with an embarrassing situation, that is, the shortage of literature materials. At that time, there was no distinction between literature, history, and philosophy and the concept of literature in the modern sense had not yet been fully established. As an important proposition of poetry education in the Zhou Dynasty, “elegance” originated from the natural cognition of the ancestors, then gradually acquired the ideological attribute, and finally became a standard of stylistic division or even an artistic proposition. In the Zhou Dynasty, the system of rites and music developed from basic song and dance and witchcraft etiquette. These elements were integrated into one and applied to clan tribes in ancient times. As a result, they are inextricably linked to the rise and collapse of clan tribes. The aesthetic implications of Zhou Dynasty poetics, as a crucial component of aesthetic research, can more clearly show the evolution of the aesthetic style.

Based on the text emotion analysis technology in DL (deep learning), this paper is devoted to the analysis of aesthetic implication in Zhou Dynasty poetics and the important role of this thinking in the formation of the overall aesthetic thinking style in ancient China and even in modern China. The main contributions of this paper are as follows: (1) This paper hopes to downplay the differences between disciplines, reveal the aesthetic changes of aesthetic implication in Zhou Dynasty poetics through the research and analysis of Zhou Dynasty poetics, and thus, show the nonrich connotation of Zhou Dynasty's formal beauty thought and its important position in China's formal beauty thought. (2) In this paper, the method based on feature fusion is selected to judge the emotional tendency, and the feasibility of applying DL in the analysis of aesthetic implication of Zhou Dynasty poetics is explored. On this basis, several optimization schemes are put forward to improve the accuracy of emotional tendency judgment.

## 2. Related Work

### 2.1. Related Research on Poetics of the Zhou Dynasty

Since the Han Dynasty, Confucianism has been regarded as a classic, and later, scholars have shown great interest in the study of Zhou Dynasty's poetic system and the spirit of rites and music. Some works and studies have strong historical stage characteristics, while others are practical. Sugar et al. put forward that the confluence of etiquette and law began at the end of the Warring States period, which was mainly manifested in two aspects: ideology and system [3]. Holcombe pays attention to the comprehensive application of traditional literature, field archaeology, and ancient writing materials and expounds some theoretical problems of etiquette [4]. Wai-Ming pays attention to the elaboration and deep excavation of the concept of rites and customs and has a very comprehensive and systematic research on the structural significance of various rites and customs and rites and music culture in the Zhou Dynasty [5].

The Zhou Dynasty is divided into two stages: “Western Zhou” and “Eastern Zhou.” The Zhou Dynasty is an important historical transition period in ancient China, and it is a period when the slavery society went from maturity and prosperity to decline and extinction. Therefore, at this stage, people's ideological and aesthetic concepts have also undergone great changes. Drège put forward the “meaningful form,” thinking that Chinese characters, bronze ornamentation, and architectural art are the combination of literature and quality. It is unique in that it pays great attention to the realistic investigation of artworks [6]. Wilkinson and Endymion pointed out that the Zhou Dynasty produced the embryonic form of the ethical aesthetic view focusing on the harmony and unity between people and society and believed that the core of aesthetics was implemented in the cultivation of the theme moral sentiment, and achieving the harmony and unity between individuals and society was the utilitarian requirement of aesthetics [7]. Fraser believed that the Zhou Dynasty was a period when tangible productivity in human material production and intangible experience science in human spiritual production went hand in hand. Therefore, the whole social foundation of slavery collapsed and the superstructure and ideology including aesthetic art underwent earth-shaking changes [8].

### 2.2. Research on Text Emotion Analysis Based on DL

The use of DL in natural language processing is growing, and the DL models that go along with it have been shown to perform well in a variety of tasks. In order to assess and extract the useful elements from a massive amount of data, the DL multilayer neural network topology mimics the functioning of the human brain. It is possible to think of the features taken from DL as a higher-level abstraction of the initial text emotional data, making them useful for completing some challenging abstract recognition tasks.

Sailunaz and Alhajj put forward a method of constructing distributed word vectors by using the neural network. After mapping word vectors to low-dimensional space, the distance unit is used to measure the similarity between words [9]. Yang et al. proposed to use the CNN (convective neural network) to analyze the text sentiment of sentences [10]. In the model, multiple filters are used to scan adjacent word vectors, and then, the feature vector representation of sentences is obtained through pooling operation, and then, the text sentiment analysis is carried out. Li et al. incorporated emotional polarity information into the loss function of the neural network model to get the word vector with emotional information [11]. In order to cope with text sentiment analysis, Tocoglu et al. used the RNN (recurrent neural network) and recurrent neural tensor network models, which perform well at both predicting the sentiment polarity of single sentences and fine-grained sentiment analysis of sentences [12].

Almeida et al. use the CNN to model and solve the problem of emotion classification. Rn has a good effect on processing information containing time series data, so it is often applied to natural language processing tasks [13]. Liu et al. used the CNN neural network algorithm to model the feature information existing in the text data and then to deal with the emotion classification problem and achieved good results [14]. Zeng et al. put forward a thesaurus-based algorithm to solve the problem of emotional tendency. This algorithm adopts the bootstrapping strategy, and its emotional tendency ultimately depends on the sum of emotional tendency scores of all emotional words in a sentence [15]; Dang et al. put forward the strategy of goal dependence, considering the influence of the context on Weibo's information emotion. The main realization methods are goal dependence and situational awareness. The goal dependence method refers to judging emotion according to syntactic features, while the situational awareness method is classified by considering the related tweets of each tweet [16].

## 3. Methodology

### 3.1. Poetry Text Preprocessing Method

In the history of aesthetic development, according to archaeological research, China's aesthetic consciousness sprouted about 18,000 years ago in the “caveman” period. Since the birth of mankind, the exploration of the essence of beauty has never stopped. Humans also regard “beauty” as the highest realm of lifelong pursuit. Beauty can only come from social practice, and it is the perceptual manifestation of people's essential power. This process is subjective and dynamic, but a subjective image of the objective world, not a general reflection but a subjective, universal, advanced, and social reflection; it is not a passive reflection nor a blind and intuitive imitation but a positive and active reflection.

He is the founder of Confucianism, a great thinker, politician and educator in Chinese history, and an outstanding musician. He initiated private school running and actively advocated music education. “Ritual music” has a long history in China. Primitive people have long used rites and music for religious sacrifices, offering sacrifices to God, offering sacrifices first, offering gifts to God, and entertaining God. We can also find the records of the ritual and music activities of the primitive ancestors from other ancient documents. This can be said to be the embryonic form of Chinese ritual and music culture. In the impression of the primitive ancestors, they merged with their own subjective feelings and the primitive ancestors naturally gave their subjective feelings to the objective water. In the process of poetry expression, subjectivity and objectivity were naturally combined.

The etiquette system of the Zhou Dynasty should conform to a certain birthright status as well as morality, so the Zhou Dynasty people had to seek an appropriate and “appropriate” between them. This kind of “appropriate” is born in the system and manifested in life. That is, propriety should be moderate, people's appearance should be appropriate, and etiquette ceremony should be honest and do what one can. Studying the aesthetic culture of the Zhou Dynasty, we are more willing to explore the aesthetic pursuit of “propriety” contained in the external form of rites. Therefore, we can take “propriety” as an aesthetic category and discuss the aesthetic pursuit of propriety “propriety” in the Zhou Dynasty from the perspective of its connotation and external form. The development of productive forces in the Zhou Dynasty also made people more and more aware of the great power of “human beings” and started the ideological emancipation trend of paying attention to and pursuing “beauty.” The widespread use of iron tools marks a great breakthrough and development of social productive forces, and it is also the premise foundation of the prosperous economy and the emergence of a hundred schools of thought in the Warring States period.

The study of artificial neural networks [17, 18] is where the idea of DL came from. It is made up of multilayer nonlinear arithmetic units, with each subsequent layer receiving its input from the output of the previous layer. Effective feature representation information can be derived from a vast number of input data after multilayer connection. Text sentiment analysis can be broken down into three categories based on the level of text granularity: text sentiment analysis, sentence sentiment analysis, and word sentiment analysis. DL models have been shown to have superior results in numerous sectors as a result of the extension of the data scale, increase in processing power, and ongoing algorithm optimization. Word models are created using neural networks.

Text preprocessing is a method of formatting text, which needs to process unstructured or semistructured data such as word segmentation, sentence segmentation, and stop word removal, in order to extract the required information from rough original data. This section discusses the improved text segmentation method. The main idea of the improvement is that firstly, the maximum matching method is used to roughly segment the text, then, the hidden Markov model is used to mark the part of speech of the segmented words, and then, the part of speech marking and segmentation results are evaluated to get the best segmentation results.

The goal of part-of-speech tagging is to reduce the amount of calculation required and increase the algorithm's operating efficiency by removing words that are unnecessary or contribute little to the text's content. For the hidden Markov model, assuming that the result set of word segmentation after word segmentation is *W* and the part-of-speech state set is *T* and assuming that words are independent of each other, the probability of segmenting *W* is as follows:

(1) $$\begin{array}{c} P\left(W\right)=\overset{m}{\prod }P\left(w_{j}\right). \end{array}$$

The conditions for splitting *W* in the part-of-speech state *T* are as follows:

(2) $$\begin{array}{c} P\left(W\left|T\right.\right)=\overset{m}{\prod }P\left(w_{j}\left|t_{j}\right.\right). \end{array}$$

The poetry of the Zhou Dynasty is incredibly unstructured, has no set framework, and uses a free form. To implement the mapping from discrete text to real number space in this work, GloVe is used. In other words, the concept of statistical probability of word cooccurrence is introduced on the basis of the skip-gram method. This method learns word vectors based on the statistical information of global word cooccurrence, thus combining the statistical information with the method of the local context window. In order to save additional information about the cooccurrence of text words, the GloVe model creates a rough matrix of the vocabulary cooccurrence matrix. We have the following calculation formula:

(3) $$\begin{array}{c} X_{i}=\overset{V}{\underset{k=1}{\sum }}X_{i,k},\\ P_{ik}=\frac{X_{i,k}}{X_{i}}, \end{array}$$

where *X*_*i*_ represents the sum of words appearing in a row of matrix words *i*; *V* represents the total amount of words in the dictionary; it indicates the number of times that the *X*_*i*,*k*_ word *j* and the word *k* appear together in a fixed window in the training corpus; *P*_*ik*_ indicates the probability that the word *k* appears in the fixed window in the word *i*.

As an LSTM network version, the GRU (gate recurrent unit) can also address the issue of long-term reliance brought on by RNN networks. As a result, it is currently among the most common network structures [19]. In contrast to GRU, which has two gating structures (an update gate and a reset gate), LSTM has three: an input gate, a forgetting gate, and an output gate. It is the unit structure diagram of GRU, as seen in Figure 1.

The update gate, represented by *Z*_*t*_, is used to regulate how much the state data from the previous instant is incorporated into the current state. The amount of state information from the previous instant that is brought in increases with the update gate's value. *r*_*t*_ stands for the reset gate. The amount of information from the previous moment written depends on how big the reset gate is.

The vectorization technology is the most important data processing method in natural language processing tasks, which directly affects the results of most text analysis tasks [20]. Word vector technology maps text vocabulary sequences into continuous vector space, which is different from the previous word feature representation in that word embedding can not only better represent the feature information of text semantics but also uniformly distribute the vector expressions of words with similar meanings.

AM (attention mechanism) is used to characterize the correlation between words in a text sentence and the output result, indicating the importance of each word in sentence *x*_*i*_ and its corresponding label *y*_*i*_. During the experiment, the formal expression of the text features obtained by AM is as follows:

(4) $$\begin{array}{c} s_{i}=f_{\text{att}}\left(x_{ij},y_{i}\right),\;1\leq i\leq m,1\leq j\leq n, \end{array}$$

where *x*_*i*_ represents a text sentence representation in the input data, *y*_*i*_ represents the emotion classification label corresponding to the input data sentence, and *f*_att_ represents a three-layer feedforward neural network structure.

### 3.2. Analysis of Aesthetic Implication of the Poetry Text in the Zhou Dynasty Based on DL

Some of the color descriptions in “The Book of Poetry” are simple descriptions of objective things, while more color choices contain profound aesthetic and cultural implications, and the same color often has several different symbolic meanings. Yellow in “The Book of Poetry” roughly expresses three meanings, namely, power, decay, and longevity. The symbol of power comes from people's worship of land, while the meaning of decay and longevity comes from people's association with natural phenomena. It is the color of green vegetation, and people think of people from things, so the most beautiful and vibrant age stage in life is also called “green.” The color of vegetation is also the easiest to arouse people's feelings, compared with the warmth of love conveyed by red. Personally, the agreement between the two sides in “The Book of Poetry” shows that the emotion of the lyrical hero is in harmony with the color picture and artistic conception shown in the poem. Although this color landscape lacks romantic fantasy and rich luxury, it is simple and full of fresh spiritual breath, which is in the same strain as the folk song nature of “The Book of Poetry.”

Music culture has always been dominated by the display of poetry and music in the elegant music of the court. The development of songs and music in the Zhou Dynasty is based on sound, singing, and harmony. On this basis, music and dance performances and instrumental accompaniment are added. Songs, music, and dance together constitute the overall structure of music in the Zhou Dynasty. Because folk songs are handed down from mouth to mouth, their songs and lyrics are kept in the memory of folk singers in the form of sound. Once they are written and incorporated into the dynasty music system by music institutions, they will inevitably enter the writing system according to the requirements of the ritual and music system. The development of Chinese music in “The Book of Poetry” has been very perfect, and the fusion of poetry and music has reached the peak of poetry and music culture. When it depicts the shape and appearance of the development of a social song and music culture in words, it also shows the brilliant achievements of poetic civilization in the Zhou Dynasty. Therefore, to a certain extent, we can say that the development and inheritance of poetry and music should promote and help each other. “The Book of Poetry” with song and music culture actually has very important historical and social significance.

Dance is an example of an action-based kind of material with an independent value, whereas music is an example of a sound-based material with an independent value. Poetry then takes on a form composed of words with a meaning of its own. Mourning poems are elegies compiled by the poet with his heart and soul, taking feelings as the classics and death as the latitude. They are one of the closest and most direct literary forms to express death. Therefore, the consciousness of death is an integral part of people's life consciousness and it is the ultimate reflection on people's tragic fate and the essence of human existence. It contains the attitude towards death and belief in life, respect for the personality of the deceased, and cherishing of the value of life.

Text analysis mainly includes sentiment analysis, text classification, and sentiment tendency prediction. It mainly relies on the emotional tendency of words in the text and the context of words for emotional analysis. On the basis of extracting text features by text vectorization, it classifies the features by the machine learning algorithm. When the amount of text is large, the perceptron model with a multilayer structure can be constructed by the DL method and the problems of text classification, sentiment analysis, and so on can be solved by the calculation model obtained by training data and circular learning.

This research suggests a CNN-LSTM poetic aesthetic implication analysis approach based on the idea of self-attention to address the issues with the classic Chinese short-text emotion analysis model that semantic information is easy to lose and emotional information may be overlooked. The goal of the attention model's process is to mimic human brain attention. When observing something, the human brain will provide specific attention to some aspects of it for a predetermined amount of time while temporarily disregarding aspects in other areas. This is a method for the human brain to make rational use of resources. AM is the process of weighting the target data. According to the task type, different weighting processes are carried out on each part of the model input. AM was first applied to the research of computer vision.

For the IL (input layer), word vectors trained by Word2Vec are used and then input into the CNN-LSTM joint model. Then, the output of the joint model is weighted and summed by self-attention and finally input into the Softmax classifier, so as to realize the emotion classification of the text, as shown in Figure 2.

Use Word2Vec to convert the comment text processed in the previous step from vocabulary to quantification. Firstly, a word vector dictionary is established, so that each text word has a unique trained word vector corresponding to it. For the text words that do not appear, the word vectors are randomly initialized. Because AM gives particular attention to select features, it can give more weight to significant features in sentences when using a DL model to train feature representation, which increases the precision of emotion categorization. After performing the aforementioned actions, the feature representation of the input text sentence data can be generated by simultaneously establishing several filters to extract the features from the input text data.

The word vectors in the text vocabulary are spliced to generate a sentence-level word vector matrix, as shown in formula (5).

(5) $$\begin{array}{c} S_{ij}=V\left(w\left(1\right)\right)⊕V\left(w\left(2\right)\right)⊕\cdots ⊕V\left(w\left(i\right)\right). \end{array}$$

*w*(1), *w*(2), ⋯, *w*(*i*) represents the text vocabulary; *V*(*w*(1)), *V*(*w*(2)), ⋯, *V*(*w*(*i*)) represents the word vector corresponding to the text vocabulary; *S*_*ij*_ represents the word vector matrix of the *j*th sentence spliced by *i* word vectors; ⊕ represents the splicing operation of word vectors.

The convolution kernel *w* ∈ *R*^*hk*^ in convolution operation indicates that a window contains *h* words to generate a new feature. For example, the *i*th to *i* + *h* − 1th words are the features *c*_*i*_ generated by a window, as shown in formula (6).

(6) $$\begin{array}{c} c_{i}=f\left(w\cdot x_{i:i+h-1}+b\right). \end{array}$$

*b* ∈ *R* is the bias term, *f* is the nonlinear activation function, and tan*h* function is adopted.

Two HL (hidden layers) run from the front end and the back end of IL, so that the information of the context before and after the input statement can be considered, where *h*_*t*_, *g*_*t*_ is the neuron node corresponding to HL and the parameter solving equation is as follows:

(7) $$\begin{array}{c} h_{t}=f\left(U_{h}x_{t}+W_{h}h_{t-1}+b_{h}\right),\\ g_{t}=f\left(U_{g}x_{t}+W_{g}g_{t-1}+b_{g}\right). \end{array}$$

AM is a system to achieve effective resource allocation. The fundamental tenet of AM is that important components of the input data are given more weight while less weight is given to other items. To improve the overall model's optimization outcome and model accuracy, use AM to calculate the probability distribution of attention for various sections and then obtain the various degrees of influence that each portion of the input has on the output result. For text sentiment analysis, the characteristic expression of the text is calculated as follows:

(8) $$\begin{array}{c} u_{t}=\tan h\left(w_{s}h_{t}+b_{s}\right),\\ y_{i}=\text{softmax }\left(W_{i}d_{ijt}+b_{i}\right), \end{array}$$

where *W*_*i*_ represents the weight matrix from the dense layer to the output layer; *b*_*i*_ represents the corresponding bias; *d*_*ijt*_ represents the output vector of the dense layer at time *t*.

## 4. Experiment and Results

In order to prove the validity of the CNN-LSTM aesthetic implication analysis model of Zhou Dynasty poetics based on the thought of self-attention, it is verified by several different groups of experiments. This paper selects the public IMDB movie review dataset. There are two categories of datasets, positive and negative, which represent positive and negative, respectively. Text sentiment analysis experiments based on DL in this paper are all designed on the open-source DL library Keras, which is a highly modular neural network library written in the Python language.

The ReLU function is employed as the activation function in the experiment for the network structure model suggested in this paper, and many groups of convolution kernels are used for training. Convolution kernel window sizes are set to 2, 3, and 4, there are 100 convolution neurons in each filter and 300 HL neurons, and Softmax is used to classify the output layer. The experimental comparative analysis is presented in Table 1 to demonstrate the efficacy of the CNN-LSTM aesthetic implication analysis model of Zhou Dynasty poetics based on the concept of self-attention.  Figure 3 displays the outcomes of data visualization.

It can be seen that the overall performance of this model is better than that of the other three comparison models for the quantification of evaluation indexes. The accuracy and F1 of this paper are 93.362% and 90.886%, both of which are higher than other models, and the LSTM model has also achieved good classification results. It shows that the model in this paper is superior to the other three models under the same situation of introducing AM at the same time and can achieve better classification effect.

As can be seen in Figure 4, for other models in the experiment, the overall change is an upward trend, while the overall fluctuation of this model is small, and the fluctuation range is small and at the lowest value. For other models in the experiment, the overall change is an upward trend, while the overall fluctuation of this model is small, and the fluctuation range is small and at the lowest value.

According to Figure 5, CNN's 50 times text classification effect is slightly better than RNN's classification effect. The main reason is that it can always obtain the most important influence factors in the text in convolution and pooling processing and obtain high-order features by combining features layer by layer.

It can be seen that their classification effect is obviously inferior to that of LSTM. In addition, according to the curve of the 50 times classification effect, the classification effect of the above four algorithms is relatively stable and the classification effect of this algorithm is more stable. When the size of the text library is within a certain range, it is a competitive text classification algorithm. The number of training sets randomly generated in the above text database totaled 50 times, and 50 training sets were obtained. The above four algorithms are applied to these 50 training sets and then tested by the corresponding test sets. The average time of each algorithm is shown in Table 2.

It can be concluded that the RNN needs the most running time, mainly because the input of the current neuron in the RNN is influenced by the output of the front and back neurons in the sequence, and the adjustment and training of parameters need to take into account the parameter values of the front and back neurons in the sequence.

This algorithm takes the least time, mainly because this method uses the existing Word2Vec word vector feature weighting to get the text vector, which saves the process of the training neural network, and there is no complicated neural network training process.

In order to get the word vector representation of the input text data in the model, this paper selects Chinese corpus from Wikipedia as the training sample and makes an experiment by using the word vector method mentioned. The context size is set to 5, and if any words are not in the pretrained word vector, they are represented by random initialization. Finally, the effect is verified by comparing the selected datasets and the experimental results are shown in Figure 6.

From the experimental results in Figure 6, it can be seen that the classification accuracy of the model is the highest when the word vector with 150 dimensions is selected and the accuracy begins to decrease when the queen is increased. Therefore, this experiment selects the distributed word vector with 150 dimensions for the next experiment.

Setting different percentage of dropout values will have certain influence on the performance of the sentiment analysis system. Therefore, in this experiment, the change of sentiment analysis performance of the LSTM neural network is observed by changing the value of dropout under the condition that other parameters are unchanged, as shown in Figure 7.

According to the experimental findings, the model's sentiment analysis performance first increases and subsequently drops when the dropout value grows. The evaluation index values all increase to their maximum when the dropout value is 0.5, and the macroaverage accuracy rate is 95.006%. The model's training time will also be impacted by the dropout value, though. The model's training time decreases as the dropout value increases. As a result, in the real world, choosing the dropout value should take the model's training time into account in addition to the evaluation index value.

## 5. Conclusion

At the end of the Shang Dynasty, the slave society had gradually matured and the accumulation of certain social capital made people have higher and higher requirements for life. People began to notice the important role of ornaments. The Western Zhou Dynasty was the peak of the ritual and music system. Under the background of the ritual and music system, the concept of formal beauty in the Western Zhou Dynasty flourished. It is not difficult to see that the poetic thoughts and aesthetic standards of the Zhou Dynasty, which were conceived in it, are characterized by the combination of poetry and thinking. Zhou Dynasty poetics appear in our daily communication as a spiritual form with aesthetic significance, which can make people get along and communicate with each other from a perceptual point of view, and pull the spiritual distance between people. The research on text analysis using the DL neural network is booming, which provides a powerful tool for deep semantic analysis of the text. Based on the analysis of the emotional polarity of texts and the similar classification of texts, this paper constructs a CNN-LSTM aesthetic implication analysis model of Zhou Dynasty poetics based on the thought of self-attention. The research results show that the overall performance of this model is better than that of the other three comparison models for the quantification of evaluation indexes. The accuracy and F1 of this paper are 93.362% and 90.886%, respectively, which are higher than other models. The comparative analysis of numerical experiments shows that this method can effectively classify texts, and its running efficiency is within an acceptable range.

## Figures and Tables

**Figure 1:** GRU unit structure diagram.

**Figure 2:** Model diagram of CNN-LSTM based on self-attention.

**Figure 3:** Comparison data visualization.

**Figure 4:** Change trend of loss in different models.

**Figure 5:** Accuracy of different model classification.

**Figure 6:** The influence of vector dimensions on results.

**Figure 7:** Change trend of macroaverage accuracy corresponding to different dropout values.

**Table 1:** Comparison results of different models.

Model	Accuracy	Recall	F1
CNN	84.282	89.37	87.865
LSTM	87.33	90.28	85.985
RNN	86.587	89.176	88.314
Our	93.362	91.147	90.886

**Table 2:** Comparison of average running time of different models.

Model	Run time (s)
CNN	1369.71
LSTM	1553.28
RNN	2130.61
Our	1025.14

## Data Availability

The data used to support the findings of this study are available from the corresponding author upon request.
